# Action Intention Understanding EEG Signal Classification Based on Improved Discriminative Spatial Patterns

**DOI:** 10.1155/2021/1462369

**Published:** 2021-11-23

**Authors:** Xingliang Xiong, Hua Yu, Haixian Wang, Jiuchuan Jiang

**Affiliations:** ^1^Key Laboratory of Child Development and Learning Science of Ministry of Education, School of Biological Science & Medical Engineering, Southeast University, Nanjing 210096, Jiangsu, China; ^2^Department of Cardiology, The First Affiliated Hospital of USTC, Division of Life Sciences and Medicine, University of Science and Technology of China, Hefei 230001, Anhui, China; ^3^School of Information Engineering, Nanjing University of Finance and Economics, Nanjing 210003, Jiangsu, China

## Abstract

**Objective:**

Action intention understanding EEG signal classification is indispensable for investigating human-computer interactions and intention understanding mechanisms. Numerous investigations on classification tasks extract classification features by using graph theory metrics; however, the classification results are usually not good.

**Method:**

To effectively implement the task of action intention understanding EEG signal classification, we proposed a new feature extraction method by improving discriminative spatial patterns.

**Results:**

The whole frequency band and fusion band achieved satisfactory classification accuracies. Compared with other authors' methods for action intention understanding EEG signal classification, the new method performs more satisfactorily in some aspects.

**Conclusions:**

The new feature extraction method not only effectively avoids complex values when solving the generalized eigenvalue problem but also perfectly realizes appreciable classification accuracies. Fusing the classification features of different frequency bands is a useful strategy for the classification task.

## 1. Introduction

Action intention understanding is that a subject determines the direct goal behind an object's motor behaviors [1, 2], which lays a solid foundation for some activities, such as social interaction [3] and language learning [4]. Recently, many people have investigated action intention understanding [5–13]. Some of them focused on neuro mechanism analysis [5, 6, 14], while others pay close attention to signal classification [7–12, 14]. It is important to note that we principally address action intention understanding EEG signal classification in this article. An ideal classification result is extremely important for enriching user experiences in real life. For instance, the brain-computer interface (BCI) [9–12] highly depends on classification accuracies.

To acquire satisfactory classification accuracy for brain signals with action intention understanding, many advanced approaches have been proposed in recent years [5, 12, 14]. However, the experimental results of these approaches are not ideal and are usually lower than 60% [12, 14]. Most of these advanced approaches adopt graph theory metrics to extract classification features. Some previous studies noted that graph thresholding is prone to losing useful information [9, 10], while the lost information may enhance the classification ability. Recently, Zhang et al. [14] found that action intention understanding closely correlates with several special components (e.g., N170-200 and P400-700) in a brain network research. Liao et al. [15] proposed a novel algorithm that utilizes discriminative spatial patterns (DSP) to extract classification features to effectively classify the brain signals of movement imagery. Their experimental results indicate that the DSP is useful for extracting efficient classification features. However, complex values easily occur in DSP when calculating the generalized eigenvalue problem solution.

Therefore, in this study, we propose a new feature extraction method by modifying the DSP algorithm in special EEG components. The raw EEG signals are first preprocessed with Neuroscan and EEGLAB [16]. Then, we extract some time series fragments in special components N70, P120, N170-P200, P300, and P400-700 and combine them. Then, we use the DSP to calculate the projection vector. To further investigate the selection of the most useful classification features, we use circulation iteration to search the optical feature combination based on the data from the previous step. Finally, we use the *k*-nearest neighbor (KNN) classifier to carry out a binary classification task for action intention understanding EEG signals in five frequency bands (delta, theta, alpha, beta, and whole frequency band) and a fusion band (the combination of the five frequency bands).

The main contribution of this study is that the new feature extraction method perfectly avoids complex values when solving the generalized eigenvalue problem in the DSP. Furthermore, we found that feature extraction, feature selection, and frequency band fusion strategies are extremely effective for action intention understanding EEG signal classification.

## 2. Methodology and Materials

### 2.1. Participants

Referring to the experience of the BCI competition in single-trial classification of motor imagery [15], we also used three participants (one male and two females; aged 23–25 years, mean ± SD: 23.67 ± 1.33; physiology and psychology were healthy; right-handed) to implement the experimental task in this research. Because we mainly classify action intention understanding EEG signals based on trial level, hence, a small amount of participants does not cause the lack of generality of the proposed method.

Before the EEG signal collection experiment, all participants were first asked to read an experimental informed consent file and then sign a contract. When finishing the EEG signal collection experiment, all the participants received some compensation. This study was approved by the Academic Committee of the School of Biological Sciences and Medical Engineering, Southeast University, China.

### 2.2. Experimental Paradigm

In this study, our experimental paradigm is inspired by Ortigue et al.'s study [2].  Figure 1 presents out the overview of the experimental paradigm.  Figure 1(a) demonstrates three kinds of action intention stimuli (Ug is the intention of drinking water, Tg is the intention of moving a cup, and Sc denotes that only simply touches the cup but without any specific intention) used in this paper, Figure 1(b) presents out an example about the stimulation process in a single trial, and Figure 1(c) shows an illustration to explain what is the action intention understanding. More specific details of the experimental paradigm are shown in references [9, 10, 17].

### 2.3. EEG Data Collecting and Preprocessing

In EEG signal collection, the electrical equipment was Neuroscan 4.3, 64 channels, international 10–20 system, and 500 Hz sampling frequency. Each action intention stimulus condition contained 98 trials. Hence, every participant had 294 trials in this study.

For the raw EEG data of the three participants, ocular processing and re-reference were first completed with Neuroscan. Channel selection (60 electrodes were retained; the layout of the electrodes is shown in Figure 2), initial filtering (whole frequency band: 1–30 Hz), segmentation, baseline correction, and artefact deleting (signals at −75∼75 *μ*V were retained, i.e., the trial of which voltage signals between −75 and 75 *μ*V was retained and otherwise removed as artefact. The final trial numbers of the three participants were 68, 72, 71; 97, 96, 98; and 97, 96, 98, respectively) were then finished in the EEGLAB [16]. Four subfrequency bands (delta, theta, alpha, and beta) were finally extracted with the Butterworth filter.

### 2.4. Special Components Extraction and Combination

Recently, Zhang et al. [14] found that action intention understanding closely correlates with several special components, such as N70 and P120. Therefore, we first extract the N70, P120, N170-P200, P300, and P400-700 components and then combine these special components to obtain new time series that are more useful for classifying EEG signals with action intention understanding. For the N70, P120, and P300, we selected five sample points around the N70, P120, and P300 moments, respectively. For the N170-P200 and the P400-700, we selected multiple sample points in the time sections N170-P200 and P400-700, respectively. All the sample points that are chosen from the special components are recombined as a new matrix. It is worth mentioning that combining the special components can not only effectively delete redundant information but also improve computing efficiency.

### 2.5. Improved Discriminative Spatial Pattern

For a *N* × *T* single trial EEG data *X*_*j*_(*i*), where *N*, *T*, *i*, *j* are the number of electrodes, number of time points, trial ordinal number, and stimulus condition ordinal number, respectively, the mean of single-trial EEG signals in a category condition is written as

(1) $$\begin{array}{c} M_{j}=\frac{1}{n_{j}}\sum_{i=1}^{n_{j}}X_{j}\left(i\right), \end{array}$$

where *n*_*j*_ denotes the number of trials in the *j*th class condition. Thus, within-class scatter matrix *S*_*W*_ is defined as

(2) $$\begin{array}{c} S_{W}=\sum_{j=1}^{K}S_{j}, \end{array}$$

where

(3) $$\begin{array}{c} S_{j}=\sum_{i=1}^{n_{j}}\left(X_{j}\left(i\right)-M_{j}\right){\left(X_{j}\left(i\right)-M_{j}\right)}^{T}. \end{array}$$

And *K* is the number of class conditions (in this study, *K*=3). Hence, between-class scatter matrix *S*_*B*_ is calculated as

(4) $$\begin{array}{c} S_{B}=\sum_{j=1}^{K}n_{j}\left(M_{j}-M\right){\left(M_{j}-M\right)}^{T}, \end{array}$$

where

(5) $$\begin{array}{c} M=\frac{1}{n}\sum_{i=1}^{n}X\left(i\right), \end{array}$$

is the mean of all single-trial EEG signals.

Assume that there is a projection matrix *W*_1_ that can maximize the between-class scatter and simultaneously minimize the within-class scatter; therefore, we can obtain the projections of *S*_*W*_ and *S*_*B*_ as follows:

(6) $$\begin{array}{c} {\tilde{S}}_{W}=W_{1}^{T}S_{W}W_{1},\\ {\tilde{S}}_{B}=W_{1}^{T}S_{B}W_{1}. \end{array}$$

Then, the Fisher linear discriminative rule is

(7) $$\begin{array}{c} J\left(W_{1}\right)=\frac{\left|{\tilde{S}}_{B}\right|}{\left|{\tilde{S}}_{W}\right|}=\frac{\left|W_{1}^{T}S_{B}W_{1}\right|}{\left|W_{1}^{T}S_{W}W_{1}\right|}. \end{array}$$

where |*∗*| is determinant. To make (7) successfully realize the maximal value, the optimal projection *W*_1_ can be obtained by solving the following generalized eigenvalue problem:

(8) $$\begin{array}{c} S_{B}w_{d}=\lambda_{d}S_{W}w_{d}, \end{array}$$

where *λ*_*d*_ and *w*_*d*_ are the eigenvalue and column vector of the projection matrix *W*_1_, respectively. Formula (8) can be rewritten as follows:

(9) $$\begin{array}{c} S_{W}^{-1}S_{B}w_{d}=\lambda_{d}w_{d}. \end{array}$$

However, complex values easily occur when solving the above equation. If appear complex values when solve the generalized eigenvalue, it could not compute the project matrix as the real values, and then it could not obtain the classification features. In the signal classification of the experiment, all classification features need be real values. Liao et al. [15] solve this problem with singular value decomposition.

In this study, we design a new method to solve the generalized eigenvalue problem. For the single-trial EEG time series matrix (*X*_*j*_(*i*)) combined by the special components N70, P120, N170-P200, P300, and P400-700, we reshape the matrix as a vector. Equation (9) can be written as

(10) $$\begin{array}{c} S_{W}^{-1}\sum_{j=1}^{K}n_{j}\left(M_{j}-M\right){\left(M_{j}-M\right)}^{T}w_{d}=\lambda_{d}w_{d}. \end{array}$$

Notably, (*M*_*j*_ − *M*)^*T*^*w*_*d*_ and *λ*_*d*_ are scalars that only correlate with value size. Hence, these two scalars can be combined as a constant coefficient

(11) $$\begin{array}{c} \mu =\frac{{\left(M_{j}-M\right)}^{T}w_{d}}{\lambda_{d}}. \end{array}$$

Then, the generalized eigenvalue problem in (10) is equivalent to the following formula:

(12) $$\begin{array}{c} w_{d}=S_{W}^{-1}\sum_{j=1}^{K}n_{j}\left(M_{j}-M\right)\mu . \end{array}$$

Because we only consider the projection direction, the size of the constant coefficient *μ* has no effect on feature extraction. Thus, the formula in (12) can be rewritten as follows:

(13) $$\begin{array}{c} w_{d}^{*}=S_{W}^{-1}\sum_{j=1}^{K}n_{j}\left(M_{j}-M\right). \end{array}$$

It is noteworthy that we reshaped the raw time series matrix before solving the generalized eigenvalue problem; hence, we reshape the eigenvector *w*_*d*_^*∗*^ again to obtain the projection matrix *W*_1_. Finally, we transform the signals combined by the special components into a new feature space as follows:

(14) $$\begin{array}{c} Z\left(i\right)=W_{1}{}^{T}X\left(i\right)+\Delta , \end{array}$$

where Δ=−*W*_1_^*T*^*M* is a deviation. After obtaining the *Z*(*i*) in each trial, we then complete the feature extraction task.

### 2.6. Classification

To further select the most useful classification feature from the feature space that is created by the improved discriminative spatial pattern, we add features into the training dataset one by one in the process of classification until the classification accuracy reaches its peak. In this study, the classifier is *k*-nearest neighbor (KNN), and the parameter *k* is set to 3. To train the classification model more effectively, we used a 5-fold cross-validation strategy to train the classifier, and to obtain a more feasible classification result, we calculated the mean of 10 cross-validations as the average classification accuracy.

The whole procedure of our new method is shown in Figure 3. There are three indispensable steps for the new method. First, extracting and combining the special components proved to be closely correlated with action intention understanding by Zhang et al. [14] which can effectively delete most of the redundant information that is useless for the classification task. Second, reshaping the special component matrix into a vector is an important step that can reduce data from 2D space to 1D space. Third, transforming the generalized eigenvalue problem into calculating projection direction is the key step in the novel method that can perfectly avoid complex values.

## 3. Results

### 3.1. Classification Accuracies

Figure 4 presents the classification results on different frequency bands. From the two subfigures at the bottom of Figure 4, we can see that both the 1–30 Hz frequency band and fusion band obtain more satisfactory classification accuracies than the other four frequency bands. The highest average classification accuracies are close to 70%. Additionally, sub2 performs better than both sub1 and sub3 in these two significant frequency bands. Notably, sub2 does not always perform the best in the other four frequency bands.

To estimate the classification results more effectively, we provide detailed numerical values of four commonly used evaluation metrics (average classification accuracy (ACC), standard deviation (SD), sensitivity (SEN), and specificity (SPE)) in machine learning. Because our best experimental results are achieved on the whole frequency band and fusion band, we only show the estimations on these two important bands.  Table 1 shows the estimation details of the classification results. From the numerical values of the four classical estimation metrics, especially the sensitivity and specificity, we can see that our classification results are robust and reliable.

### 3.2. Comparisons with Previous Methods

To further estimate our new method, we provide comparisons with previous studies [12, 14].  Table 2 shows the average experimental accuracies of the different approaches.

Zhang et al.'s study only shows the classification results on the binary classification task Ug-vs-Sc, of which the highest average classification accuracy was 58.2% in EEG + fNIRS signals [12]. Our new method outperforms their method and achieves a 64.67% average classification accuracy on the Ug-vs-Sc task. It is noteworthy that our new method is 9.67 percentage points higher than Zhang et al.'s method under the same conditions (EEG signal conditions). Compared with Zhang et al.'s study [14], our new method is nearly 10 percentage points lower than their method on the Tg-vs-Sc task. However, our new method is 13.8 percentage points higher than their method on the Ug-vs-Tg task. For the classification results on the Ug-vs-Sc task, there is no obvious difference between the new method and the old method.

## 4. Discussion

To investigate whether the features extracted by our new method are useful, we implement action intention understanding EEG signal classification on five frequency bands (delta, theta, alpha, beta, and whole frequency band) and a fusion band (combining the features from the other five frequency bands). The classification is a binary classification that has three styles (Ug-vs-Tg, Ug-vs-Sc, and Tg-vs-Sc). From Figure 4 and Table 1, we know that our new method successfully extracts the useful classification features. The good classification accuracies indicate that the improved DSP finds the correct projection direction, which is the key factor in the DSP algorithm [15].

For the comparison in Table 2, both Zhang et al.'s and Zhang et al.'s studies extract classification features by graph theory metrics [12, 14], which easily lose some useful information in the process of network binarization. Some previous studies [9, 10] have addressed this point. Therefore, it may lead to some poor classification accuracies. The new method is basically based on the DSP algorithm, which extracts classification features from the time series and does not exhibit binarization; i.e., it does not have information loss. The proposed method is nearly 10 percentage points lower than Zhang et al.'s study [14] on the Tg-vs-Sc task. As for this result, we think the mainly reason is that our new method has its shortage in recognizing the abnormal action behavior. On the Tg-vs-Sc task, both action intentions Tg and Sc are more abnormal than the action intention Ug. However, our new method has its merit in recognizing normal action behavior. For instance, the new method obtains 63.8% average classification accuracy on the Ug-vs-Tg, which outperforms Zhang et al.'s [14] study.

The most important contributions of this study are mainly reflected in several aspects. First, the new feature extraction method perfectly avoids complex values [15] when solving the generalized eigenvalue problem in the DSP algorithm. Furthermore, introducing the special components closely correlated with action intention understanding into the DSP algorithm is a new idea that is different from some previous studies on DSPg the special components proved to be closely correlated with action intention understanding by that extract features from whole time series [15, 18, 19]. Finally, fusing classification features from different frequency bands and adding the classification features into the training dataset one by one to achieve the most satisfactory experimental results is an extremely important strategy.

Objectively speaking, there are also some limitations to our study. For instance, some studies [13, 20] point out that the CSP is prone to be influenced by noise and is sensitive to parameters, such as specific EEG time window used, operational frequency band, and selected channels, which may produce suboptimal results. In order to solve this problem, Jin et al. [21] propose a new feature selection method that based on the L1-Norm and Dempster–Shafer theory. It is noteworthy that the DSP algorithm is similar to the CSP; hence, the DSP might also be easily affected by the noise and parameters. In a recent research, Wang et al. [22] obtain some satisfactory classification results that combine the movement-related cortical potential (MRCP) and event-related desynchronization (ERD) features which are extracted by discriminative canonical pattern matching (DCPM) and the CSP, respectively. The principle of the DCPM algorithm correlates with the DSP. Therefore, if we combine our new method with the CSP to extract classification feature, it might obtain a more satisfactory classification result.

## 5. Conclusion

In summary, our new method demonstrates some advantages. It can be introduced into other research fields, such as emotion recognition, alcohol addiction, and motor imagery. Although the classification accuracies of our new method are better than some other methods, the new method still needs to be improved in practical application. Considering its limitations, we will further explore how to extract more effective features for the action intention understanding EEG signal classification in the future.

## Figures and Tables

**Figure 1:** Experimental paradigm. (a) Three kinds of action intention stimuli (Ug, Tg, and Sc) used in this study, (b) the stimulation process along with time axis in a trial, and (c) an illustration used to explain what is the action intention understanding [17].

**Figure 2:** Layout of the 60 channels selected in this study.

**Figure 3:** Overview of the novel method.

**Figure 4:** Classification accuracies on different frequency bands. The fusion band denotes combining the features from the five frequency bands. Sub1, sub2, and sub3 are the three participants.

**Table 1:** Classification estimation metrics.

EM	SUB	Fusion band			1–30 Hz		
		UT	US	TS	UT	US	TS
ACC	sub1	60.57	64.32	59.34	60.57	59.04	59.34
	sub2	68.42	68.27	58.83	68.42	68.27	56.42
	sub3	62.41	61.41	60.45	60.52	61.41	60.45

SD	sub1	14.22	11.67	10.41	14.22	15.14	10.41
	sub2	10.84	9.78	10.93	10.84	9.78	10.16
	sub3	11.22	10.98	10.84	10.46	10.98	10.84

SEN	sub1	60.08	59.21	69.04	60.08	62.03	69.04
	sub2	69.23	76.09	57.22	69.23	76.09	56.42
	sub3	58.67	56.21	56.38	59.18	56.21	56.38

SPE	sub1	60.94	71.73	50.59	60.94	57.11	50.59
	sub2	67.11	59.93	61.12	67.11	59.93	56.84
	sub3	66.90	66.24	64.95	63.13	66.24	64.95

The EM, SUB, UT, US, and TS in the second row denote the estimation metric, subject, Ug-vs-Tg, Ug-vs-Sc, and Tg-vs-Sc, respectively. The ACC, SD, SEN, and SPE in the first column are the average classification accuracy, standard deviation, sensitivity, and specificity, respectively.

**Table 2:** Comparisons with different methods.

Reference	Approach	Signal	Task	Classifier	Accuracy
Zhang et al. [12]	Binarized brain network (based on time series during task and phase synchronization and Pearson correlation algorithms) metric features	EEG	Ug-vs-Tg	SVM	#
			Ug-vs-Sc		55.00%
			Tg-vs-Sc		#
		fNIRS	Ug-vs-Tg	SVM	#
			Ug-vs-Sc		51.60%
			Tg-vs-Sc		#
		EEG + fNIRS	Ug-vs-Tg	SVM	#
			Ug-vs-Sc		58.2%
			Tg-vs-Sc		#

Zhang et al. [14]	Binarized brain network (based on ERP components and WPLI algorithm) metric features	EEG	Ug-vs-Tg	SVM	50.00%
			Ug-vs-Sc		64.83%
			Tg-vs-Sc		69.67%

**This paper**	**Improved DSP**	**EEG**	**Ug-vs-Tg**	**KNN**	**63.80%**
			**Ug-vs-Sc**		**64.67%**
			**Tg-vs-Sc**		**59.54%**

The Ug-vs-Tg, Ug-vs-Sc, and Tg-vs-Sc denote binary classification. The symbol “#” represents there is no classification task. fNIRS is the functional near-infrared spectroscopy.

## Data Availability

All data included in this study are available upon request by contact with the corresponding author.

## References

[1] Gallese V., Rochat M., Cossu G., Sinigaglia C. (2009). Motor cognition and its role in the phylogeny and ontogeny of action understanding. *Developmental Psychology*.

[2] Ortigue S., Sinigaglia C., Rizzolatti G., Grafton S. T. (2010). Understanding actions of others: the electrodynamics of the left and right hemispheres. a high-density EEG neuroimaging study. *PLoS One*.

[3] Hari R., Kujala M. V. (2009). Brain basis of human social interaction: from concepts to brain imaging. *Physiological Reviews*.

[4] Casteel M. A. (2011). The influence of motor simulations on language comprehension. *Acta Psychologica*.

[5] Catur C. (2015). Understanding intentions from actions: direct perception, inference, and the roles of mirror and mentalizing systems. *Consciousness & Cognition*.

[6] Ge S., Ding M., Zhang Z., Lin P., Gao J., Wang R. (2017). Temporal-spatial features of intention understanding based on EEG-fNIRS bimodal measurement. *IEEE Access*.

[7] Liu H., Zheng W., Sun G., Shi Y. Action understanding based on a combination of one-versus-rest and one-versus-one multi-classification methods.

[8] Pereira J., Ofner P., Schwarz A., Sburlea A. I., Müller-Putz G. R. (2017). EEG neural correlates of goal-directed movement intention. *NeuroImage*.

[9] Xiong X., Yu Z., Ma T., Wang H., Lu X., Fan H. (2020a). Classifying action intention understanding EEG signals based on weighted brain network metric features. *Biomedical Signal Processing and Control*.

[10] Xiong X., Yu Z., Ma T., Luo N., Wang H., Lu X. (2020). Weighted brain network metrics for decoding action intention understanding based on EEG. *Frontiers in Human Neuroscience*.

[11] Zhang D., Yao L., Chen K., Monaghan J. (2019). A convolutional recurrent attention model for subject-independent EEG signal analysis. *IEEE Signal Processing Letters*.

[12] Zhang Z., Yang Q., Leng Y., Yang Y., Ge S. (2016). Classification of intention understanding using EEG-NIRS bimodal system. *International Computer Conference on Wavelet Active Media Technology & Information Processing*.

[13] Zhang Y., Wang Y., Jin J., Wang X. (2017). Sparse Bayesian learning for obtaining sparsity of EEG frequency bands based feature vectors in motor imagery classification. *International Journal of Neural Systems*.

[14] Zhang L., Gan J. Q., Zheng W., Wang H. (2017). Spatiotemporal phase synchronization in adaptive reconfiguration from action observation network to mentalizing network for understanding other’s action intention. *Brain Topography*.

[15] Liao X., Yao D., Wu D., Li C. (2007). Combining spatial filters for the classification of single-trial EEG in a finger movement task. *IEEE Transactions on Biomedical Engineering*.

[16] Arnaud D., Scott M. (2004). EEGLAB: an open source toolbox for analysis of single-trial EEG dynamics including independent component analysis. *Journal of Neuroscience Methods*.

[17] Xiong X., Ge S., Lu X., Wang H. Power spectral density features for classifying action intention understanding EEG signals.

[18] Tang Q., Wang J., Wang H. (2014). L1-norm based discriminative spatial pattern for single-trial EEG classification. *Biomedical Signal Processing & Control*.

[19] Wang H., Xu J. (2011). Local discriminative spatial patterns for movement-related potentials-based EEG classification. *Biomedical Signal Processing & Control*.

[20] Samek W., Kawanabe M., Muller K.-R. (2014). Divergence-based framework for common spatial patterns algorithms. *IEEE Reviews in Biomedical Engineering*.

[21] Jin J., Xiao R., Daly I., Miao Y., Wang X., Cichocki A. (2020). Internal feature selection method of CSP based on L1-norm and Dempster-Shafer theory. *IEEE Transactions on Neural Networks and Learning Systems*.

[22] Wang K., Xu M., Wang Y., Zhang S., Chen L., Ming D. (2020). Enhance decoding of pre-movement EEG patterns for brain–computer interfaces. *Journal of Neural Engineering*.

